# Understanding the Critical Role of Glycolysis-Related lncRNAs in Lung Adenocarcinoma Based on Three Molecular Subtypes

**DOI:** 10.1155/2022/7587398

**Published:** 2022-02-07

**Authors:** Peng Cao, Bo Zhao, Yajie Xiao, Shan Hu, Kangle Kong, Peng Han, Jiaqi Yue, Yu Deng, Zhikun Zhao, Dongfang Wu, Lu Zhang, Fan Li

**Affiliations:** ^1^Department of Thoracic Surgery, Tongji Hospital, Tongji Medical College, Huazhong University of Science and Technology, No. 1095 Jiefang Avenue, Wuhan, 43000 Hubei Province, China; ^2^Department of Clinical Translational Medicine, Yucebio Biotechnology Co., Ltd, Yantian District, Shenzhen, Guangdong Province, 4th Floor, Phase I, Dabaihui Center, No. 2002, Shenyan Road, Haishan Street, Yantian District, Shenzhen, China; ^3^Department of Oncology, Tongji Hospital, Tongji Medical College, Huazhong University of Science and Technology, No. 1095 Jiefang Avenue, Wuhan, 43000 Hubei Province, China

## Abstract

**Background:**

Glycolysis is closely associated with tumor progression, but the roles of lncRNAs in glycolysis have not been comprehensively investigated in lung adenocarcinoma (LUAD). This study is aimed at studying the possible mechanisms of glycolysis-related lncRNAs in tumor development and providing a guidance for targeted therapy.

**Methods:**

Unsupervised consensus clustering was used to identify molecular subtypes. Gene enrichment analysis was applied to screen important pathways involved in tumor progression. A series of immune analysis was performed to assess immune infiltration. Critical transcription factors (TFs) interacting with lncRNAs were selected by Pearson correlation analysis. A first-order partial correlation analysis was implemented to identify critical lncRNAs with prognostic significance.

**Results:**

Three molecular subtypes (C1, C2, and C3) were identified with distinct overall survival. Three subtypes showed differential immune infiltration, and C3 subtype was the optimal for immunotherapy treatment. Ten lncRNA-TF pairs among four glycolysis-related lncRNAs (FTX, LINC00472, PSMA3-AS1, and SNHG14) and six TFs (FOXP1, SP1, MYC, FOXM1, HIF1A, and FOS) were involved in tumor progression. We identified four critical glycolysis-related lncRNAs significantly associated with prognosis.

**Conclusions:**

This study identified three molecular subtypes that could guide personalized therapy. The four-lncRNA prognostic model can serve as an indicator for predicting prognosis or early screening of lung adenocarcinoma patients. The current results improve the understanding of the relation between lncRNAs and glycolysis.

## 1. Introduction

Lung cancer is a leading cause of cancer death worldwide, and lung adenocarcinoma (LUAD) is the most common primary lung cancer. Smoking, including primary or secondary exposure to tobacco smoke, is a main risk factor for developing lung cancer. The incidence and mortality showed a decline since 1980s; according to the global cancer statistics in 2020, 2,206,771 new cases (11.4% of total new cases of cancer) were diagnosed, and 1,796,144 deaths (18.0% of total cancer deaths) of lung cancer were reported [1]. 5-year survival of lung cancer is lower than 15% largely because most of the patients are already advanced at the time of diagnosis [2–4]. However, an early screening and diagnosis of lung cancer is currently a great challenged.

Lung adenocarcinoma belongs to non-small-cell lung cancer (NSCLC) and has replaced squamous cell lung cancer as the most prevalent type of NSCLC in the past two decades [5]. Advances in detecting gene mutations and genome variations have discovered genetic alternations as one of the mechanisms contributing to NSCLC development. For example, mutations in *p53* gene occur in over half of NSCLC cases, and epidermal growth factor receptor gene (*EGFR*) and Kirsten rat sarcoma viral oncogene homolog (*KRAS*) mutations are associated with worse clinical outcome [2]. Tyrosine kinase inhibitors such as erlotinib or gefitinib could prolong 5-year survival of metastatic NSCLC patients with *EGFR* mutation to 14.6% as compared with lower than 5% of nontreated patients [6]. However, only a small number of patients can benefit from tyrosine kinase inhibitors. Therefore, mechanisms of tumorgenesis for lung cancer are needed to be explored to increase early diagnose rate and facilitate personalized therapies.

In the recent years, long noncoding RNAs (lncRNAs) have been found to play critical roles in tumorgenesis, tumor immune microenvironment, and tumor metastasis in lung adenocarcinoma as well as in many other cancer types [7]. For example, LUADT1 is high expressed in LUAD and can promote cancer cell proliferation through interacting with SUZ12 and mediating the trimethylation of H3K27 at the promoter region of p27 [8]. DGCR5 is also upregulated in LUAD, and downregulation of DGCR5 is associated with favorable prognosis [9]. Studies have discovered various lncRNA signatures for predicting prognosis of LUAD from different aspects; for example, researchers have identified prognostic lncRNAs from lncRNA-ceRNA network [10] and also developed a four-lncRNA signature with immune features [11]. These newly identified signatures provide guidance to predict prognosis and contribute to a better understanding of the mechanisms related to lncRNAs in LUAD.

In this study, we associated glycolysis with lncRNAs to further reveal the mechanisms of tumor development in LUAD. Highly active glycolysis in cancer cells produces more energy for cancer cell proliferation and could therefore serve as a target for cancer treatment [12, 13]. lncRNAs are regulators in activating or suppressing expression of genes involved in glycolysis, and a series of lncRNAs, such as LINC00857 [14], LINC01123 [15], NORAD [16], and so on, have been discovered to function to regulate glycolysis in LUAD. In the present study, we identified a number of glycolysis-related lncRNAs and explored three molecular subtypes with clinical value for guiding personalized immunotherapy. Importantly, based on a lines of bioinformatics analysis, we discovered the possible roles and mechanisms of lncRNAs for regulating glycosis in LUAD. This study developed a four-lncRNA signature related to glycolysis for predicting prognosis of LUAD. The current findings emphasized the critical role of lncRNAs and provided possibilities for discovering therapeutic drugs based on glycolysis-related lncRNAs.

## 2. Materials and Methods

### 2.1. Data Information and Preprocessing

RNA-seq data and expression profiles of LUAD samples were obtained from The Cancer Genome Atlas (TCGA, https://portal.gdc.cancer.gov/) database and Gene Expression Omnibus (GEO, https://www.ncbi.nlm.nih.gov/geo/) database. TCGA-LUAD dataset containing RNA-seq data was downloaded from TCGA, while samples without clinical information were excluded. Ensembl ID was converted to gene symbol. 485 samples in TCGA-LUAD dataset were finally included. GSE31210 [17] and GSE72094 [18] datasets were downloaded from GEO. Samples of GSE cohort were selected if survival time was longer than 30 days but shorter than 15 years. Probes without value or mapped to multiple genes were excluded. Median value was taken when multiple probes were mapped to one gene. Totally 226 and 386 samples from in GSE31210 and GSE72094 datasets remained data preprocessing, respectively. The workflow of the overall study is shown in Figure 1.

### 2.2. Acquisition of lncRNA Expression Profiles

GSE31210 and GSE72094 datasets were used for reannotation to obtain lncRNA expression profiles. Fasta file of probe sequence was downloaded from GPL570 and GPL15048 chip platform, and that of transcription reference sequence was downloaded from GENCODE (https://www.gencodegenes.org/human/). SeqMap [19] tool was used to blast probe sequence and reference sequence under nonmismatch condition. Then, GTF (gene transfer format) file downloaded from GENCODE [20] was used to distinguish lncRNA expression profile from mRNA expression profile in TCGA-LUAD, GSE31210, and GSE72094 datasets.

### 2.3. Identification of Glycolysis-Related lncRNAs

Genes related to glycolysis (hallmark glycolysis pathway) were downloaded from MSigDB database [21] (https://www.gsea-msigdb.org/gsea/msigdb/). Glycolysis score of each sample in three datasets was calculated by single sample gene set enrichment analysis (ssGSEA) using GSVA R package [22]. Pearson correlation analysis between glycolysis score and lncRNAs was conducted. Glycolysis-related lncRNAs were selected when ∣correlation coefficient | >0.3 and *p* < 0.05.

### 2.4. Unsupervised Consensus Clustering for Identifying Molecular Subtypes

Unsupervised consensus clustering was applied to construct consensus matrix and subtyping samples based on the expression of glycolysis-related lncRNAs using ConsensusClusterPlus R package [23]. PAM algorithm was used, and distance metric of “1 - Pearson correlation coefficient” was set to perform 500 times of bootstraps. Each bootstrap contained 80% samples as training group. Cluster number *k* = 2 to 10 was used to calculate consensus matrix and cumulative distribution function (CDF) to confirm the optimal clusters.

### 2.5. Enrichment Analysis of Functional Pathways

GSEA was conducted to enrich hallmark genes downloaded from Molecular Signatures Database (MSigDB, https://www.gsea-msigdb.org/gsea/msigdb/) database. To assess the function of glycolysis-related lncRNAs, ClusterProfiler R package was used to annotate functional pathways in TCGA-LUAD dataset [24].

### 2.6. Immune Analysis of Three Molecular Subtypes

CIBERSORT [25](https://cibersort.stanford.edu/) was performed to visualize the enrichment of immune cells. Estimation of Stromal and Immune cells in MAlignant Tumours using Expression data (ESTIMATE) was performed to calculate stromal score, immune score, and ESTIMATE score of the samples [26]. The TIDE [27] software (http://tide.dfci.harvard.edu/) was employed to predict the immune response of three molecular subtypes to immunotherapy.

### 2.7. Assessment of TF Activity

TF activity was assessed using a method from Garcia-Alonso et al. [28]. Firstly, gene expression of each sample was normalized by CDF [22]. Then, TF activity was approximated as a function of the collective mRNA levels of its targets using analytic Rank-based Enrichment Analysis (aREA) in VIPER R package [29]. Relative TF activity was estimated by normalized enrichment score (NES). NES = 0 was the cut-off to define relative high or low TF activity. ANOVA was performed to compare the TF activity among the three molecular subtypes. TFs with differential activity were screened by *p* < 0.05.

### 2.8. A First-Order Partial Correlation Analysis

A first-order partial correlation analysis was implemented to assess correlation among glycolysis-related lncRNAs, glycolysis score, and glycolysis-related genes. The glycolysis score was assumed to be *x*, and expression of glycolysis-related genes was assumed to be *y*. The first-order partial correlation between *x* and *y* conditioned on lncRNAs was:

(1) $$\begin{array}{c} {\text{r}}_{x\text{ylncRNA}}=\frac{{\text{r}}_{x\text{y}}‐{\text{r}}_{x\text{lncRNA}*}{\text{r}}_{\text{ylncRNA}}}{\sqrt{\left(1‐{\text{r}}_{x\text{lncRNA}}^{2}\right)*\left(1‐{\text{r}}_{\text{ylncRNA}}^{2}\right)}} \end{array}$$

### 2.9. Construction of a Prognostic Model

Four glycolysis-related lncRNAs identified by the first-order partial correlation analysis were used to construct a prognostic model. Univariate Cox regression analysis was performed to calculate correlation coefficients between the four lncRNAs and overall survival. The prognostic model was defined as risk score = (beta *i* × exp *i*), where *i* represents lncRNAs, exp *i* represents the expression of lncRNAs, and beta *i* represents the correlation coefficients. Samples were classified into high-risk and low-risk group according to the cut-off of *z* − score = 0.

### 2.10. Copy Number Variation (CNV) Analysis and Mutation Analysis

We downloaded from GDC (https://portal.gdc.cancer.gov/) the MuTect2 [30] software processed Simple Nucleotide Variation dataset and CNV dataset; we used the R package maftools (version 2.8.05) to evaluate mutation characteristics, compared mutations and copy number differences in different molecular subtype using chi-square tests, and visualized them using the function oncoplot in R package maftools [31].

## 3. Results

### 3.1. Constructing Molecular Subtypes of LUAD Based on Glycolysis-Related lncRNAs

Three datasets of TCGA-LUAD, GSE31210, and GSE72094 were included to screen lncRNAs related to glycolysis activity. A total of 3940 lncRNAs in TCGA-LUAD dataset, 379 in GSE31210, and 586 in GSE72094 were identified to be associated with glycolysis activity (Figure 2(a)). 37 of the lncRNAs coexisted in all three datasets, and they were selected for further analysis. In TCGA-LUAD dataset, 485 samples were included for consensus clustering using ConsensusClusterPlus R package. According to the CDF and relative change under CDF curve, cluster number *k* = 3 was determined to classify samples into three groups (Figures 2(b) and 2(c)). Therefore, a consensus matrix was visualized, and three molecular subtypes of C1, C2, and C3 were identified when *k* = 3 (Figure 2(d)).

To validate the effectiveness of the clustering, the relations between molecular subtypes and overall survival (OS), subtypes and glycolysis score were assessed in three datasets. Survival plots showed that three molecular subtypes had distinct OS, with the most favorable OS in C3 group and the worst OS in C1 group across all three datasets (TCGA-LUAD: *p* = 0.00039, GSE31210 and GSE72094: *p* < 0.0001; Figures 2(e)–2(g)). In addition, we calculated glycolysis score based on glycolysis-related genes by ssGSEA in three datasets. Different glycolysis scores in three molecular subtypes were observed, and the C1 group had the highest glycolysis score, but the C3 group had the lowest glycolysis score (*p* < 0.0001, Figures 2(h)–2(j)). The above results proved that the subtyping system could effectively classify LUAD samples into three molecular subtypes significantly associated with prognosis and glycolysis score. Based on the results, we speculated that LUAD prognosis was associated with glycolysis score.

### 3.2. Three Molecular Subtypes Were Closely Associated with Clinical Stages

Next, we analyzed the relation between molecular subtypes and clinical features. In TCGA-LUAD dataset, the C3 group showed a high proportion of age ≥ 60, and the C1 group had a low proportion of age < 60 (Figure 3(a)). Female patients consisted of a larger percent than male patients in the C3 group, but no significant gender difference was shown among three groups (Figure 3(b)). In relation to stage, mild stages including T1 stage, N0 stage, M0 stage, and stage I accounted for the highest proportion in the C3 group when compared with other two groups (Figures 3(c)–3(f)), which was consistent with the previous result of the most favorable prognosis of the C3 group (Figure 2(e)). For smoking status, current smokers composed the largest proportion in the C3 group, while the proportion of nonsmokers was similar among the three groups (Figure 3(g)). We also assessed the clinical features in other two datasets, GSE31210 and GSE72094. Age and gender were not significantly related to molecular subtypes, but the tendency of stage distribution was correspondent with the results in TCGA-LUAD dataset (Supplementary Figure S1A-F). However, no significant difference of smoking status was detected in three groups (Supplementary Figure S1G).

### 3.3. Differences of Genome Variation and Gene Mutation Patterns among Molecular Subtypes

Genome variations were measured to assess whether there was a correlation between genome stability and molecular subtypes through adopting five dimensionalities including aneuploidy score, homologous recombination defects, fraction altered, number of segments, and tumor mutation burden. C1 and C2 groups showed similar scores of aneuploidy score, fraction altered, number of segments, and tumor mutation burden, but the C2 group had more homologous recombination defects than the C1 group (Figure 4(a)). In all these five aspects, the C3 group obtained the lowest score, suggesting the least genome variations of the C3 group compared with other two groups (Figure 4(a)). Simultaneously, the relation between glycolysis score and genome stability was analyzed by Pearson correlation analysis. The result demonstrated that glycolysis score was positively associated with genome variations, indirectly proving that the C3 group with a high glycolysis score had higher genome variations (Figure 4(b)).

In the case of gene mutations, the C1 group had the largest number of gene mutations, while the C3 group had the smallest number of mutations (Figure 4(c)). The top 10 mutated genes were listed and *TP53*, *TTN*, and *RYR2* accounted for a majority of mutations. Missense mutation, nonsense mutation, and multihit mutation (different combinations of multiple genetic mutations) were common mutation types. Small-scale copy number variations (CNVs) of genes were also evaluated in three groups. Interestingly, the C2 group had obviously high percentage of both gain or loss of CNVs (Figure 4C). *CDKN2A* had the most number of loss of CNVs in all three groups but largely in the C1 group. *ACTRT3* contained about 20% gain of CNVs in the C1 group, while the highest number of CNV amplification in the C2 group was detected in *AGO2*.

### 3.4. Analyzing Functional Pathways of Molecular Subtypes Based on Hallmark Genes

Functional pathways of three datasets were enriched based on hallmark genes using GSEA, and FDR < 0.05 was selected to screen differentially enriched pathways between C1 and C3 subtypes. The data revealed that 29 pathways with 27 activated and 2 suppressed were enriched in TCGA-LUAD dataset (Figure 5(a)). In GSE31210 and GSE72094 datasets, 26 and 18 pathways were enriched, respectively. 13 pathways related to cell cycle, immune response, and oncogenesis, including E2F targets, G2M checkpoint, MYC targets, MTORC1, glycolysis, epithelial mesenchymal transition (EMT), unfolded protein response, DNA repair, mitotic spindle, interferon gamma response, hypoxia, and spermatogenesis pathways, were coenriched in all three datasets (Figure 5(a)). Furthermore, enrichment scores of enriched pathways were compared between C1 and C3 groups and C2 and C3 groups in three datasets, as shown in radar plots (Figures 5(b)–5(d)). Obvious high enrichment scores of the pathways were found in the C1 and C2 groups when compared with the C3 group, indicating that the activation of these pathways may be associated with unfavorable prognosis. In addition, the C1 group had relatively higher enrichment score than the C2 group, which further supported our speculation.

### 3.5. Differential Immune Infiltration of Three Molecular Subtypes

To some extent, immune infiltration can decide the degree of tumor progression, and high infiltration of cytotoxic T cells can efficiently kill tumor cells. Therefore, we obtained a series of marker genes related to different types of immune cells from a previous research [32] and calculated enrichment score of LUAD samples grouped by molecular subtypes through ssGSEA in three datasets. Three datasets showed similar distribution of immune cells in three molecular subtypes, and the majority of immune cells were differentially enriched (Figure 6(a)). Notably, the C2 group displayed low immune infiltration than the C1 and C3 groups, while the C3 group had higher infiltration of immune cells, such as cytotoxic cells, T cells, dendritic cells (DCs), and mast cells than the C1 group (Figure 6(a) and Supplementary Figure S2). Moreover, ESTIMATE measurement was applied to further evaluate the immune infiltration of three molecular subtypes. In TCGA-LUAD and GSE72094 datasets, the C2 group presented the lowest enrichment score of stromal score, immune score, and ESTIMATE score (Figure 6(b)), which was in accordance with the result of Figure 6(a). However, the C1 and C3 groups showed comparable enrichment score of the three terms in TCGA-LUAD and GSE72094 datasets, and no significant difference was observed in GSE31210 dataset (Figure 6(b)). To further examine the difference of immune infiltration between C1 and C3 groups, hierarchical clustering was performed to classify the samples into low- and high-immune infiltration. The results demonstrated that the C3 group had a higher immune infiltration than the C1 group, although part of the C1 group also showed a high enrichment of immune cells (Supplementary Figure S3).

### 3.6. Difference Responses to Immunotherapy of Three Molecular Subtypes

We then evaluate the prediction ability of three molecular subtypes for guiding immunotherapy based on the expression of immune checkpoints and TIDE analysis. A total of 18 immune checkpoints were screened to be differentially expressed among three subtypes (Figures 7(a)–7(c) and Supplementary Figure S4). A majority of immune checkpoints were high expressed in the C1 group, while the C2 group showed a low expression level of most immune checkpoints. Of 18 differentially expressed immune checkpoints, CD276, HAVCR2, and TNFSF4 were detected in all three datasets, and CD244, CD274, CD80, ICOS, IDO1, LAG3, and VISTA were identified in two datasets, and the rest 8 immune checkpoints were only identified in one dataset (Figure 7(d)). These immune checkpoints, especially CD276, HAVCR2, and TNFSF4 showing similar distribution in three datasets, may serve as potential targets for immunotherapy. In addition, we used TIDE to predict immune response to immunotherapy, with a high TIDE score representing high possibility of immune escape. The result showed that the C3 group had the lowest TIDE score among three molecular subtypes in all three datasets (Figures 7(e)–7(g)), indicating that the C3 group may develop a favorable prognosis after immunotherapy.

### 3.7. The Aberrant Expression of Transcriptional Factors Was Associated with Glycolysis-Related lncRNAs and Tumor Progression

In the previous sections, we demonstrated that glycolysis-related lncRNAs were associated with prognosis, tumor- and immune-related pathways, and immune infiltration in LUAD patients, but the role of glycolysis-related lncRNAs play in regulating glycolysis remained unclear. It has been shown that the function of lncRNAs to act in *cis* in the nucleus and *trans* in the nucleus or cytoplasm is dependent on their subcellular localization [33]. lncRNAs can up- or downregulate gene expression level commonly through the interactions with TFs or chromatin-modifying complexes [34]. Therefore, here, we attempted to reveal possible mechanisms of glycolysis-related lncRNAs in tumor development.

A total of 37 glycolysis-related lncRNAs identified in all three datasets were selected for the following analysis. In the relation between the expression of protein-coding genes (PCGs) related to glycolysis and lncRNAs, we observed that the expressions of most lncRNAs were negatively correlated with that of PCGs (Figure 8(a)), indicating that glycolysis-related lncRNAs were possibly in negative regulation to glycolysis-related PCGs expression. Then, LncATLAS database was employed to study the localization of glycolysis-related lncRNAs, and relative concentration index (RCI) was used to quantify the localization. We found that the majority of lncRNAs localized in nucleus presented as negative (RCI < 0) accounted for 83.28% in TCGA-LUAD dataset, 63.21% in GSE31210 dataset, and 71.29% in GSE72094 dataset (Figure 8(b)). To specifically evaluate the localization of 37 lncRNAs, we included 15 types of cell lines. The data showed that most lncRNAs were highly enriched in the nucleus, which was consistent with the above results (Supplementary Figure S5).

Subsequently, we assessed the activity of TFs in three molecular subtypes according to aREA algorithm, and each sample obtained a score of TF activity. The difference of TF activity among three subtypes was analyzed in three datasets, and 46, 32, and 46 TFs with differential activity among three subtypes were screened in TCGA-LUAD, GSE31210, and GSE72094 datasets, respectively (Supplementary Table S1). Then, we analyzed the relation between these TFs and the lncRNAs localized in the nucleus. 13 TFs were identified to be negatively associated with the nuclear lncRNAs, and E2F4, FOXM1, MYC, and E2F1 TFs were all present in three datasets (Figure 8(c)). Notably, significantly negative correlation was observed in a number of lncRNA-TF pairs among lncRNAs of FTX, LINC00472, PSMA3-AS1, SNHG14, and TFs of FOXP1, SP1, MYC, FOXM1, HIF1A, and FOS (*R* ≤ −0.3, Figure 8(d)). The results suggested that the nuclear lncRNAs could interact with TFs, and these lncRNA-TF pairs may function critically in regulating glycolysis.

To analyze whether there was a difference of TF expression among three molecular subtypes, we compared the expression of 13 TFs associated with nuclear lncRNAs in TCGA-LUAD dataset. The C1 group had relatively higher expression of most TFs than other two groups (Figure 9(a)), and we also observed similar results in GSE31210 and GSE72094 datasets (Supplementary Figure S6), indicating that the upregulation of these TFs may be correlated with worse prognosis. Furthermore, we analyzed enriched pathways of these TFs, and a series of tumor-related pathways, such as PI3K-AKT signaling pathway, proteoglycans in cancer, cellular senescence, cell cycle, and small cell lung cancer, were annotated (Figure 9(b)). The above results demonstrated that glycolysis-related lncRNAs may be involved in tumor progression of LUAD through negatively regulating the expression of TFs.

### 3.8. Identification of Four Central Glycolysis-Related lncRNAs with Prognostic Significance for LUAD

First-order partial correlation was conducted among glycolysis score, the expression of glycolysis-related lncRNAs, and glycolysis-related genes to examine the key role of glycolysis-related lncRNAs in regulating glycolysis (Figure 10(a)). As a result, four lncRNAs, LINC00511, LINC00472, ADAMTS9-AS2, and LINC00968, showed a strong correlation with glycolysis score and glycolysis-related genes. Moreover, the correlation between glycolysis score and glycolysis-related genes obviously weakened when these four lncRNAs were excluded, indicating that the four lncRNAs were closely involved in glycolysis-related pathways. Then, we identified the corresponding glycolysis-related genes of the four lncRNAs and applied gene enrichment analysis to screen enriched pathways. Several pathways closely associated with tumor development were enriched, for instance, cell cycle, p53 signaling pathway, DNA replication, and mismatch repair pathways (Figure 10(b)). In addition, we compared the expression of these four key lncRNAs between primary tumor samples and adjacent cancer normal tissue in the TCGA-LUAD cohort. It can be seen that the expression of these four key lncRNAs varied significantly in both tumor and normal samples. Among them, the LINC00511 expression was significantly higher in the tumor samples than in the normal samples. However, LINC00472, ADAMTS9 AS2, and LINC00968 were significantly higher in normal tissues than in tumor samples (Supplementary Figure S7A). Similarly, the four key lncRNAs are differentially expressed in the three molecular subtypes. The expression of LINC00511 in C1 and C2 subtypes is significantly higher than that in C3 subtypes (supplementary figure S7B). Furthermore, whether these four lncRNAs could serve as predictors to evaluate prognosis for LUAD patients was assessed by calculating the correlation coefficients between the four lncRNAs and overall survival, and a prognostic model was constructed. Each sample was calculated by the prognostic model for a risk score, which was converted to *z*-score for classifying samples into high-risk and low-risk groups. In three datasets, samples were all clearly classified into high-risk and low-risk groups, suggesting that these four lncRNAs could be indicators for predicting prognosis of LUAD (Figures 10(c)–10(e)).

## 4. Discussion

Previous research has demonstrated that glycolysis is more active in cancer cells than normal cells, and that some lncRNAs have been proven to serve as promoting or suppressing roles in orchestrating glycolysis-related pathways. However, a systematical exploration on relation between lncRNAs and glycolysis has not been studied with LUAD. Therefore, this study focused on examining the possible mechanisms of lncRNAs for coordinating glycolysis in LUAD based on a series of bioinformatics analysis.

We first identified 37 lncRNAs significantly associated with glycolysis score (calculated based on the expression of glycolysis-related genes) and subsequently classified three molecular subtypes according to the expression of these lncRNAs. Three molecular subtypes (C1, C2, and C3) exhibited distinct overall survival and differential glycolysis score in all three datasets, where C1 subtype had the worst prognosis and the highest glycolysis score and C3 was the converse. These molecular subtypes provided a preliminary evidence that glycolysis-related lncRNAs were involved in LUAD development. In the relation between subtypes and clinical features, the proportion of mild stages such as T0, N0, M0, and stage I was higher in C3 subtype. The observation further confirmed the subtyping and critical role of glycolysis-related lncRNAs in LUAD progression.

Following the above findings, the molecular subtypes can be a basis for discovering the functional pathways critically involved in tumor development. Therefore, differentially enriched pathways between C1 and C3 subtypes were screened based on hallmark genes. Apart from glycolysis pathways, other oncogenic pathways such as E2F target, G2M checkpoint, DNA repair, MYC targets, and EMT were also identified to be highly enriched in C1 subtype. E2F target, G2M checkpoint, and DNA repair pathways are responsible to cell cycle progression and are associated with cancer progression [35–37]. We obtained information on the immune molecular subtypes of TCGA-LUAD from a previous study by Thorsson et al. [38], in which the authors classified lung adenocarcinomas into five immune molecular subtypes based on 160 different immune signatures, with the best prognosis was immune subtype C3. In addition, we compared the relationship between these five immune molecular subtypes and the three molecular subtypes we identified (Supplementary Figure S8), and the analysis showed that the immune subtype C3 subtype occupied more of the C3 molecular subtype we defined, whereas in Vesteinn Thorsson's study the immune molecular subtype C3 (inflammatory) molecularly characterised by elevated Th17 and Th1 genes, low to moderate tumor cell proliferation, lower levels of aneuploidy, and overall somatic cell copy number alterations than the other subtypes, and in terms of prognostic analysis, the C3 subtype has the best prognosis of the five immune subtype molecular subtypes, which is consistent with our molecular subtype C3 having the best prognosis, and we also found a poorer prognosis of the immune molecular subtypes C1, C2, C4, and C6 occupy more of the C1 and C2 subtypes in our study, which is also consistent with the poorer prognosis of C1 and C2.

Studies suggested that E2F target is a potential therapeutic target in lung cancer. The inhibitor HLM006474 of E2F target can reduce the viability of NSCLC cell lines [39]. Park et al. found that lncRNA-EPEL promotes lung cancer cell proliferation through activating E2F target pathway, and EPEL could be a potential target for therapeutic treatments [40]. G2M checkpoint is associated with DNA damage and genome stability, and a less efficient G2M checkpoint was proven to be significantly correlated with lung cancer risk [41]. In addition, through genotype-phenotype correlation analysis, Zheng et el. showed that polymorphisms in cell cycle and DNA repair can modulate the function of G2M checkpoint in lung cancer [41]. Compared with C3 subtype, C1 subtype demonstrated a significantly high level of genetic variations, especially *TP53* gene involved in cell cycle. A large number of copy number variations in C1 subtype will lead to high genome instability. A positive correlation between genome instability and glycolysis score was presented in this study. Apart from the mild correlation, we found a supplementary evidence that genome instability was responsible for aberrant suppression or activation of cell cycle pathways, which therefore contributed to dysregulation of glycolysis-related lncRNAs. EMT is a pivotal process that facilitates cell development and cancer progression, especially when in an active state in aggressive cancers [42]. EMT signatures are considered as indicators of unfavorable prognosis in many cancer types, including lung cancer [43, 44]. Evidence indicates that EMT can promote glycolysis and increases glycolytic dependency [45, 46], which also makes it sensible that C1 subtype with the highest glycolysis activity showed high enrichment of EMT signaling pathway.

As the subtyping was validated to be reliable, we further analyzed whether these subtypes could guide personalized therapy. Immunotherapy as a promising strategy for cancer treatment has been investigated in many cancer types and manifested satisfactory outcomes in partial clinical trials [47, 48]. Lines of immune checkpoint inhibitors (ICIs) have been tested in metastatic NSCLC, and some have been approved by the United States Food and Drug Administration (FDA), for instance, nivolumab [49], pembrolizumab [50], and atezolizumab [51]. Although patients with advanced NSCLC can benefit from these ICIs, still some are not sensitive to these drugs. In the present study, C1 and C3 subtypes showed a higher expression level of ICIs and immune infiltration than C2 subtype. Theoretically, C1 and C3 subtypes are both suitable objects for receiving immune checkpoint blockade (ICB) therapy, but TIDE analysis predicted that only C3 subtype can benefit the most from immunotherapy. We speculated that the possible reason for this result was due to the high activation of EMT in C1 subtype. Apart from the promoting role of EMT in cancer metastasis, drug resistance driven by EMT has also been recognized [52, 53]. As Thompson et al. proposed that responders to ICB in lung cancer have higher EMT signature scores than nonresponders, while higher inflammatory scores is observed in the responders [54], EMT status is a restrictive factor for ICB therapy. Therefore, C3 subtype may be the optimal object for receiving immunotherapy. The subtyping can provide a guidance for deciding personalized therapy for lung cancer patients.

Furthermore, we investigated the possible mechanism of glycolysis-related lncRNAs in modulating glycolysis and found that the majority of glycolysis-related lncRNAs had a negative relation with the expression of protein coding genes related to glycolysis, indicating a negative regulation between lncRNAs and glycolysis genes. These lncRNAs mostly localized in the nucleus, which demonstrated that they functioned the role prior to protein coding or gene transcription. We further examined the relation between lncRNAs and TFs, and significant correlations among four lncRNAs (FTX, LINC00472, PSMA3-AS1, and SNHG14) and six TFs (FOXP1, SP1, MYC, FOXM1, HIF1A, and FOS) were shown by Pearson correlation analysis.

FOXP1 is associated with prognosis of various malignant tumors, and low expression or loss of FOXP1 is predictive of poor prognosis of lung cancer [55, 56]. Hsu et al. proved that overexpression of SP1 can upregulate the expression of E-cadherin, a suppressor of metastasis, and downregulated expression level of SP1 was shown in invasive late-stage LUAD model in mice [57]. In our result, although elevated expression was observed in LUAD patients, higher expression of SP1 was shown in C1 subtypes than other two subtypes. MYC is an oncogene in many cancers and also serve as a metastatic gene in NSCLC [58]. Xu et al. found that FOXM1 can promote tumor progression through EMT, and that knockdown of FOXM1 can suppress the metastatic abilities in NSCLC cells [59]. High FOXM1 expression was also shown in C1 subtype. Overexpression of HIF1A is common in NSCLC, and it is associated with activation of angiogenic factors and a poor prognosis [60]. Consistent with the previous study, C1 subtype exhibited high expression level of HIF1A. The FOS family also plays an important role in tumorgenesis, but its overexpression results in different outcomes depending on different cancer types [61]. Collectively, the aberrant expression of six TFs was all found to be involved in tumorgenesis or tumor progression possibly through the interactions with the four lncRNAs and thus contributed to a worse prognosis of C1 subtype.

Finally, we identified four key glycolysis-related lncRNAs closely involved in oncogenic pathways such as cell cycle and p53 signaling pathway. We also proposed a four-lncRNA prognostic model with clinical significance in classifying LUAD patients into high-risk and low-risk groups. These four lncRNAs could be indicators for early screening of LUAD.

## 5. Conclusions

In conclusion, this study identified three molecular subtypes with distinct prognosis based on glycolysis-related lncRNAs and confirmed the subtyping through assessing their clinical features and genetic variations. Moreover, the subtyping could guide the personalized therapy, and C3 subtype was supposed to be the optimal group for receiving immunotherapy. The possible mechanism of glycolysis-related lncRNAs involved in tumor progression was possibly realized through interacting with the six critical TFs. Lastly, we constructed a four-lncRNA prognostic model predictive of LUAD prognosis and could serve as an indicator for LUAD patients.

## Figures and Tables

**Figure 1:** Work flow chart.

**Figure 2:** Identification of three subtypes based on glycolysis-related lncRNAs. (a) Venn plot of lncRNAs related to glycolysis in TCGA-LUAD, GSE31210, and GSE72094 datasets. Pos represents lncRNAs that are positively related to glycolysis score, while Neg represents lncRNAs that are negatively related to glycolysis score. (b) CDF curve when cluster number *k* = 2 to 10 in TCGA-LUAD dataset. (c) Relative change in area under CDF curve when *k* = 2 to 10 in TCGA-LUAD dataset. (d) Consensus matrix when *k* = 3 in TCGA-LUAD dataset. (e–g) Kaplan-Meier survival curve of three molecular subtypes (C1, C2, and C3) in TCGA-LUAD (e), GSE31210 (f), and GSE72094 (g) datasets. Log-rank test was performed. (h–j) Glycolysis score of three molecular subtypes in TCGA-LUAD (h), GSE31210 (i), and GSE72094 (j) datasets. Kruskal-Wallis test was performed. ns: no significance. ^∗∗∗∗^*p* < 0.0001.

**Figure 3:** The relation between three molecular subtypes and clinical features including age (a), gender (b), T stage (c), N stage (d), M stage (e), stage (f), and smoke status (g). ANOVA was performed.

**Figure 4:** Genomic variations and mutation patterns of three molecular subtypes in TCGA-LUAD dataset. (a) The difference of aneuploidy score, homologous recombination defects, fraction altered (the fraction of bases pairs present in the copy number profiles deviating from the baseline ploidy), number of segments (the total number of segments present in the copy number profile of each sample), and tumor mutation burden among three subtypes. Kruskal-Wallis test was performed. (b) Pearson correlation analysis between glycolysis score and genomic variations. (c) The difference of mutation patterns of the top 10 altered genes among three subtypes. ns: no significance. ^∗∗∗^*p* < 0.001, ^∗∗∗∗^*p* < 0.0001.

**Figure 5:** Enrichment analysis of functional pathways based on hallmark genes. (a) A heat map revealing the differentially enriched pathways between C1 and C3 subtypes with FDR < 0.05. NES: normalized enrichment score of C1 vs. C3. (b–d) Radar plots presenting the NES of enriched pathways of C1 vs. C3 and C2 vs. C3 in TCGA-LUAD (b), GSE31210 (c), and GSE72094 (d) datasets.

**Figure 6:** The differential immune infiltration of three molecular subtypes. (a) Estimated proportion of 24 types of immune cells in TCGA-LUAD, GSE31210, and GSE72094 datasets. aDC: active dendritic cells; iDC: immature dendritic cells; NK cells: natural killer cells; pDC: plasmacytoid dendritic cells; Tcm cells: central memory T cells; Tem cells: effector memory T cells; Tfh cells: T follicular helper cells; Tgd cells: gamma delta T cells. (b) Comparison of stromal score, immune score, and ESTIMATE score among three subtypes in TCGA-LUAD, GSE31210, and GSE72094 datasets. ANOVA was performed. ns: no significance. ^∗^*p* < 0.05, ^∗∗^*p* < 0.01, ^∗∗∗^*p* < 0.001, ^∗∗∗∗^*p* < 0.0001.

**Figure 7:** The relation between molecular subtypes and immunotherapy. (a–c) The differential expression of immune checkpoints among three molecular subtypes in TCGA-LUAD (a), GSE31210 (b), and GSE72094 (c) datasets. exprs: expression; ANOVA was performed. (d) The frequency of 18 immune checkpoints present in three datasets. Horizontal axis represents the number of times. Freq: frequency. (e–g) TIDE analysis for predicting the immune response to immunotherapy in three subtypes in TCGA-LUAD (e), GSE31210 (f), and GSE72094 (g) datasets. Kruskal-Wallis test was performed. False represents positive immune response, and true represents negative immune response. ns: no significance. ^∗^*p* < 0.05, ^∗∗^*p* < 0.01, ^∗∗∗^*p* < 0.001, ^∗∗∗∗^*p* < 0.0001.

**Figure 8:** The relation between glycolysis-related lncRNAs and TFs. (a) The correlation analysis between glycolysis-related lncRNAs and PCGs in TCGA-LUAD, GSE31210, and GSE72094 datasets. Horizontal axis represents correlation coefficients, and vertical axis represents the density of corresponding coefficients. (b) The localization analysis of glycolysis-related lncRNAs based on LncATLAS database. Positive indicates lncRNAs localize in the cytoplasm (RCI > 0), and negative indicates nucleus (RCI < 0). (c) The distribution of upregulated TFs negatively correlated with glycolysis-related lncRNAs in three datasets. Freq: frequency. (d) The Pearson correlation analysis between TFs and glycolysis-related lncRNAs in three datasets. Pairs with coefficient ≤ −0.3 and *p* < 0.05 were presented.

**Figure 9:** Analysis of possible mechanism of glycolysis-related lncRNAs regulating glycolysis. (a) The differential expression of 13 upregulated TFs negatively correlated with glycolysis-related lncRNAs in TCGA-LUAD dataset. ANOVA was performed. (b) Enriched pathways of TFs upregulated in C1 subtype in TCGA-LUAD dataset. ns: no significance. ^∗^*p* < 0.05, ^∗∗^*p* < 0.01, ^∗∗∗^*p* < 0.001, ^∗∗∗∗^*p* < 0.0001.

**Figure 10:** Identification of four glycolysis-related lncRNAs associated with prognosis. (a) A first order partial correlation analysis among glycolysis-related lncRNAs, glycolysis-related genes, and glycolysis score. Solid lines exhibit CDFs of correlation coefficients between glycolysis score and gene expression without adjustment. Dotted lines exhibit CDFs of correlation coefficients between glycolysis score and gene expression adjusted by first-order partial correlation. (b) Function analysis of genes significantly associated with four glycolysis-related lncRNAs in TCGA-LUAD dataset. Size indicates the number of genes. (c–d) Kaplan-Meier survival analysis of high-risk and low-risk groups in TCGA-LUAD (c), GSE31210 (d), and GSE72094 (e) datasets. Log-rank test was performed.

## Data Availability

The data used to support the findings of this study are included within the article.

## Abbreviations

CDF: Cumulative distribution function
CNVs: Copy number variations
DCs: Dendritic cells
EGFR: Epidermal growth factor receptor gene
EMT: Epithelial mesenchymal transition
ESTIMATE: Estimation of STromal and Immune cells in MAlignant Tumours using Expression data
FDA: The United States Food and Drug Administration
FDR: False discovery rate
GEO: Gene expression omnibus
ICB: Immune checkpoint blockade
KRAS: Kirsten rat sarcoma viral oncogene homolog
lncRNAs: Long noncoding RNAs
LUAD: Lung adenocarcinoma
MSigDB: Molecular signatures database
NES: Normalized enrichment score
NSCLC: Non-small-cell lung cancer
OS: Overall survival
PCGs: Protein-coding genes
RCI: Relative concentration index
ssGSEA: Single sample gene set enrichment analysis
TCGA: The Cancer Genome Atlas
TFs: Transcription factors.

## Supplementary Materials

Supplementary 1 Supplementary Figure S1: the relation between molecular subtypes and clinical features in GSE31210 (A-C) and GSE72094 (D-G) datasets. ANOVA was performed.

Supplementary 2 Supplementary Figure S2: the comparison of distribution of 24 immune cells between C1 and C3 subtypes. Student's *t*-test was performed. ns: no significance. ^∗^*p* < 0.05, ^∗∗^*p* < 0.01, ^∗∗∗^*p* < 0.001, ^∗∗∗∗^*p* < 0.0001.

Supplementary 3 Supplementary Figure S3: unsupervised consensus clustering for immune cell infiltration in C1 and C3 subtypes in TCGA-LUAD (A), GSE31210 (B), and GSE72094 (C) datasets.

Supplementary 4 Supplementary Figure S4: the normalized gene expression of immune checkpoints in three datasets grouped by molecular subtypes. ANOVA was performed. ns: no significance. ^∗^*p* < 0.05, ^∗∗^*p* < 0.01, ^∗∗∗^*p* < 0.001, ^∗∗∗∗^*p* < 0.0001.

Supplementary 5 Supplementary Figure S5: the localization of 37 glycolysis-related lncRNAs in 15 types of cell lines. Blue-green indicates lncRNAs localized in the nucleus, and red indicates in the cytoplasm.

Supplementary 6 Supplementary Table S1: differential TF activity among three subtypes in TCGA-LUAD, GSE72094, and GSE31210 datasets based on aREA algorithm. ANOVA was performed.

Supplementary 7 Supplementary Figure S6: the expression of 13 TFs in GSE31210 (A) and GSE72094 (B) datasets grouped by molecular subtypes. ANOVA was performed. ns: no significance. ^∗^*p* < 0.05, ^∗∗^*p* < 0.01, ^∗∗∗^*p* < 0.001, ^∗∗∗∗^*p* < 0.0001.

Supplementary 8 Supplementary Figure S7: expression difference of four lncRNAs. (A) Differential expression of four lncRNAs in cancer and adjacent tissues. (B) Expression differences of four lncRNAs in different molecular subtypes.

Supplementary 9 Supplementary Figure S8: intersection of the three molecular subtypes with the five immune molecular subtypes previously reported by Vesteinn Thorsson's et al.
